# Blockchain-Based Reversible Data Hiding for Securing Medical Images

**DOI:** 10.1155/2021/9943402

**Published:** 2021-05-07

**Authors:** Ji-Hwei Horng, Ching-Chun Chang, Guan-Long Li, Wai-Kong Lee, Seong Oun Hwang

**Affiliations:** ^1^Department of Electronic Engineering, National Quemoy University, Kinmen 89250, Taiwan; ^2^Department of Electronic Engineering, Tsinghua University, Beijing 100084, China; ^3^Department of Information Engineering and Computer Science, Feng Chia University, Taichung 40724, Taiwan; ^4^Department of Computer Engineering, Gachon University, Republic of Korea

## Abstract

Medical images carry a lot of important information for making a medical diagnosis. Since the medical images need to be communicated frequently to allow timely and accurate diagnosis, it has become a target for malicious attacks. Hence, medical images are protected through encryption algorithms. Recently, reversible data hiding on the encrypted images (RDHEI) schemes are employed to embed private information into the medical images. This allows effective and secure communication, wherein the privately embedded information (e.g., medical records and personal information) is very useful to the medical diagnosis. However, existing RDHEI schemes still suffer from low embedding capacity, which limits their applicability. Besides, such solution still lacks a good mechanism to ensure its integrity and traceability. To resolve these issues, a novel approach based on image block-wise encryption and histogram shifting is proposed to provide more embedding capacity in the encrypted images. The embedding rate is over 0.8 bpp for typical medical images. On top of that, a blockchain-based system for RDHEI is proposed to resolve the traceability. The private information is stored on the blockchain together with the hash value of the original medical image. This allows traceability of all the medical images communicated over the proposed blockchain network.

## 1. Introduction

The medical industry has been moving toward the digitized era, wherein a large amount of medical information is stored in a digital form and communicated digitally [1]. This helps in streamlining the acquisition, processing, and management of medical information and, at the same time, improving the efficiency in the medical industry. From all medical information, medical health record (MHR) is the most vital part, as it keeps all the important and private information regarding the patients and their diagnosis. MHR usually includes the patients' information like personal data, medical history, medical images, diagnosis reports, etc. Due to the booming of telemedicine technology, the exchange of medical images is becoming an important trend in the medical industry [2]. Medical image is one of the critical pieces of information in MHR that reveals a lot of sensitive information, which needs to be protected against malicious intrusion.

Traditional cryptographic algorithms can be used in protecting MHR (including medical images) effectively. For instance, Alam et al. [3] had proposed a framework for provisioning healthcare data, wherein Elliptic Curve Cryptography (ECC) and Advanced Encryption Standard (AES) are being used to encrypt the medical data. Recently, there is an increasing trend in employing reversible data hiding (RDH) techniques to embed sensitive information into medical images. RHD schemes have found some applications to the medical images, which are reported by Yang et al. [4, 5]. This shows that RDH is a promising candidate in securing medical images with the additional ability to embed sensitive information, which is not found in traditional cryptographic algorithms.

RDH is a technique that allows perfect recovery of the original plain image and the embedded data. The embedded data is usually some important or sensitive data to be hidden within the plain image. For instance, in the context of medical images, this can be the patient's personal data, diagnosis report, and summary of past medical records related to the medical images. The study [6] presented a flexible RDH scheme based on quad-tree and pixel value ordering (PVO) to exploit the similarity between neighboring pixels to hide more data. The paper [7] proposed a method that does not take the difference of the neighboring pixels in an image. Instead, they rearrange the columns/rows of the image in a way that improves the smooth regions, resulting in an increase in embedding capacity.

Recently, more attention turned toward RDH on the encrypted images (RDHEI). This is to ensure that the security and privacy of the transmitted image are being protected. Although these proposed RDHEI schemes are advanced and able to securely communicate the images and hidden data, they are still vulnerable to certain malicious activities. In particular, one can still modify the pixel values in an encrypted medical image for a malicious purpose, which should be detected. In other words, the integrity of RDHEI schemes needs to be checked, and this is still an open research problem to date. Moreover, the records of medical data communication are not properly protected, which makes the tracing and tracking of such communication a challenging issue to be resolved.

Blockchain is an emerging technology that aims to replace or compensate for the traditional centralized systems. It can be regarded as a Distributed Ledger Technology (DLT), wherein the transaction and storage of data are performed in a distributed manner. In such a way, even though there is no trust among all communicating parties, they can still trust the blockchain network. One of the key features of the blockchain is that all the data stored in the chain are connected through a cryptographic hash, which is very costly (or almost impossible) to tamper with.

Blockchain was recently applied to the healthcare system to improve security. For instance, [8] proposed Guardhealth, a decentralized blockchain system for privacy preserving and data sharing in medical industry. In this paper, our aim is to apply blockchain to improve integrity and traceability of the RDHEI scheme for protecting medical images.

An RDHEI scheme that vacates room after encryption of the cover image is proposed. The cover image is first divided into small blocks and then permuted by a permutation key. Then, each block is stream ciphered by an encryption key. The data hider vacates the embedding room and hides secret data using the histogram shifting technique. Our scheme can achieve a high embedding capacity compared to the state-of-the-art scheme by Zhang et al. [9]. A blockchain-based system is proposed to provide additional features to the proposed RDHEI scheme, which can be very useful in securing medical images. The contribution of this paper is summarized as follows:

1. This paper proposed an RDHEI scheme to embed private information into the medical images. The proposed scheme employed stream cipher to vacate more space for data embedding capacity compared to the state-of-the-art scheme proposed by Zhang et al. [9].
2. A novel blockchain-based RDHEI system was proposed, wherein the hash value is generated from the output of RDHEI and stored on the blockchain. This ensures that any attempt to tamper with the medical images can be detected easily.

The proposed system allows the user to exchange the ciphered steganography medical image (CSMI) securely with other members within the blockchain network. This is an important contribution to the medical industry as important medical information can be communicated frequently without worrying about security issues.

## 2. Background

### 2.1. Overview of Blockchain Technology

Blockchain is a distributed ledger system that is developed to work in an environment wherein the participating parties do not trust each other. In contrast to the traditional server-centric model, blockchain requires each participating node to store a copy of the ledger which records all the transactional details. Since the ledger is kept locally by all participating nodes, they can perform an audit on the transactions locally. With this feature, even though there is no trust among the participating nodes, one can still trust the consensus achieved through blockchain.

Another unique feature offered by blockchain is the introduction of a cryptographic hash to link up all the transaction records. Referring to Figure 1, all valid transactions are grouped into a block within a fixed time interval. A new hash value is generated based on these transaction details together with the hash of the previous block. Followed by this is the consensus process (e.g., Proof of Work (PoW)) to approve the transaction. During the consensus process, only the node that successfully solved the given difficult puzzle can add this block into the existing blockchain. The generation of hash in each transaction block is linked with the hash of the previous block. To modify one of the transaction records in the blockchain, one must generate a lot of valid blocks through the consensus process and overwrite the subsequent blocks. Since the PoW is a time-consuming process, it is very difficult to generate a lot of new blocks in a short time; this makes blockchain an immutable solution to many applications.

The consensus process through the PoW process in the blockchain is time consuming, which makes the transaction slow (e.g., 10 minutes for Bitcoin). Another alternative is to employ consortium blockchain, wherein a list of trusted members is predefined. In such case, a lightweight consensus process like Practical Byzantine Fault Tolerance (PBZT) [10] can be used. This allows timelier communication between the nodes within the same consortium blockchain, without sacrificing the key security features (i.e., auditability, traceability, and integrity) in the blockchain.

### 2.2. Overview of RDHEI

Many image steganography techniques have been proposed in the past in order to hide secret data in a way that the stego image appears with no difference from the cover image. To achieve this goal, only a slight modification of the pixel value is allowed, which severely limits the hiding capacity of a cover image. If we further constrain that the cover image should be perfectly recoverable [11] after the extraction of secret data, the embedding capacity is reduced to a very low level. Many reversible data hiding methods have been proposed to solve this challenging problem, which can be classified into three categories including lossless compression, histogram shifting, and pixel value differencing.

The lossless compression [12, 13] exploits redundancy of the cover image to embed data, in which the smooth images can hide more data than the complex images. Histogram shifting [14, 15] was proposed later on, wherein the data is embedded by shifting one side of a peak value in the histogram outward, leveraging the expanded extra space. Pixel value differencing is a more advanced technique [16, 17] that computes the differences of the pixel value in an image block and hides data by expanding the difference, in a way similar to the histogram shifting method. All these methods can embed secret data and recover the cover image after data extraction. The emergence of cloud services provides another possible framework, in which the data hiding operation is performed by a third party. RDHEI scheme can be used under this framework, wherein the content owner encrypts the cover image and sends it to the data hider to embed the secret data and forward it to the receiver. At the receiver end, the secret data can be extracted using the embedding key and the cover image can be reconstructed using the encryption key. In case the receiver is not authorized to acquire the secret data, he can still obtain the slightly distorted cover image using the encryption key only.

RDHEI schemes proposed in the past can be classified into two categories: vacating room after encryption (VRAE) and vacating room before encryption (VRBE). VRAE technique vacates room for embedding after the encryption. In 2008, Puech et al. [18] proposed an RDHEI scheme that applies bit substitution to embed secret data into an encrypted image. Later on, Zhang [19] proposed a separable RDH scheme, in which the receiver can extract secret data by using an encryption key and recover the cover image using a data hiding key. When the receiver has both keys, he can obtain both secret data and recover the image. VRBE is first proposed by Ma et al. [20] in 2013. By vacating embedding room before encryption, they claim that their scheme can achieve real reversibility; i.e., the data extraction and image recovery are free of any error. In 2016, Cao et al. [21] proposed a VRBE scheme based on sparse coding, in which the leading residual errors and learned dictionaries, together with the secret data, are embedded into the encrypted image. Malik et al. proposed an RDHEI scheme [22] that creates spare space using the prediction-error estimation method. The data is embedded into the most significant bits of the encrypted image. However, an additional location map is required to mark the nonembeddable pixels. RDHEI schemes can also be used to embed sensitive information into medical images. For instance, [4] had proposed a scheme to embed information into medical images through RDH and homomorphic encryption. Later on, [5] improved the scheme by proposing a novel paradigm (encrypt-then-RDH) to enhance the security of RDH over medical images.

Recently, Zhang et al. [9] proposed an interesting work along this research direction, in which they claim to achieve high embedding capacity. Referring to Figure 2, Zhang et al. [9] use additive homomorphic encryption and block permutation to encrypt the cover. The encryption and decryption formulas for homomorphic encryption are given by equations (1) and (2), respectively.

(1) $$\begin{array}{c} C=E\left(P,K\right)=\left(P+K\right)\mathrm{mod}N, \end{array}$$

(2) $$\begin{array}{c} P=D\left(C,K\right)=\left(C-K\right)\mathrm{mod}N, \end{array}$$

where *N* = 256, *K* is Key-1, and *E*(·) and *D*(·) are encryption and decryption algorithms, respectively. For each subblock, all pixels are encrypted using the same key to preserve the correlation between them. A block permutation method based on the chaotic algorithm is applied to strengthen security. An additional key sequence Key-2 is required to execute this operation. In the data embedding phase, the pixels in a subblock are classified into three sets according to their locations. For each set of pixels, a particular prediction rule is applied to measure prediction errors. Then, the histogram expansion and shifting process is used to embed secret data into the prediction errors. By controlling the embedding interval created by histogram expansion, the embedding capacity is adjustable. An embedding key Key-3 is required to store the information about embedding intervals.

This data hiding scheme suffers from some problems. First, homomorphic and block permutation encryptions of the cover image are not secure enough. The overall effect of image encryption is shifting of pixel gray level and changing of block spatial location. Secondly, the embedding key is not completely random, because it stores the parameters for data hiding, which is actually metadata for secret message extraction. The public key system could not help to share the encryption key under this scheme. The third and the most critical one is the problem of overflow. To hide the more secret data, the wider embedding interval should be expanded, and larger prediction errors exist. The encrypted pixel values may overflow the formal range of 0 to 255. To deal with the problems above, we propose a novel data hiding scheme in the following section.

## 3. The Proposed Reversible Data Hiding Scheme for Medical Images

In this section, we propose an RDHEI scheme based on stream ciphering and histogram shifting techniques. Our scheme includes three phases, namely, (1) the image encryption, (2) the data hiding, and (3) the data extraction and image decryption as shown in Figure 3. Three secret keys are involved in the proposed RDHEI scheme. *Key-I* and *Key-II* are the image encryption keys and *Key-III* is the data hiding key. The length of each key could be 64, 128, or 256 bits depending on the required security level. In the image encryption phase, the gray level cover image occupied by the content owner is firstly divided into mutually exclusive blocks of size 3 × 3. Block permutation with encryption key *Key-I* is applied to crumble the spatial relationship between image blocks. Then, stream ciphering with encryption key *Key-II* is leveraged to encrypt the image. In the data hiding phase, the data hider embeds secret data and metadata using the histogram shifting technique with *Key-III*. At the receiver end, the metadata is extracted first. With histogram rough restoration, the approximate cover image can be recovered using encryption keys *Key-I* and *Key-II*. With histogram fine restoration, the cover image can be perfectly recovered. For an authenticated receiver, a secret message can be deciphered from secret data using *Key-III*.

### 3.1. Cover Image Encryption Phase

The cover image encryption phase includes two steps: block permutation and stream ciphering. The cover image is divided into mutually exclusive blocks of size 3 × 3 first. Then, *Key-I* is applied to generate a random sequence of length equal to the number of total blocks in the image and all blocks are reordered according to the random sequence. An illustrative tiny image of 2 × 2 blocks is shown in Figure 4, where (a) is the original tiny image and (b) is the permuted image according to the random sequence 2; 3; 1; 0. After block permutation, we apply *Key-II* to generate a secret stream. Then, each image block is encrypted by

(3) $$\begin{array}{c} C=E\left(P,K\right)=K⊕P, \end{array}$$

where *K* is an 8-bit stream code truncated from the secret stream, *P* and *C* represent the input block and the cipher block, respectively, and the encryption function *E*(∙) is an Exclusive-OR operation denoted by “⊕.” All blocks are sequentially encrypted with a distinct 8-bit code segment for each. Pixels within the same block are encrypted with the same code segment; therefore, their correlation is preserved. This is an important feature for the following data embedding phase.

An illustrative example of the cover image encryption is shown in Figure 5. To simplify the representation, we use two blocks only to demonstrate the encryption operation. The two image blocks in (a) are permuted using the sequence generated by *Key-I* to obtain (b). Then, the two blocks are stream ciphered by two code segments generated by *Key-II*, individually. We take the first pixel of each block as an example. The binary codes of the first code segment and first-pixel value are 62=(00111110)_2_ and 104=(01101000)_2_, respectively. By Exclusive-OR operation, it results in (01010110)_2_=86. The code segment and first-pixel value of the second block are 193=(11000001)_2_ and 106=(01101010)_2_, respectively. It results in (10101011)_2_=171. Other pixels are calculated in the same way to get the result (c).

### 3.2. Data Embedding Phase

The data embedding process for the data hider is as shown in Figure 3. The preprocessing for each block in the encrypted image is an internal Exclusive-OR operation given by

(4) $$\begin{array}{c} g_{i}=c_{i}⊕c_{c},\;i=1,2,\ldots ,8, \end{array}$$

where *c*_*c*_ is the center pixel value of a block, *c*_*i*_ is a pixel value around the center pixel as shown in Figure 6(a), and *g*_*i*_ is its corresponding output pixel value as shown in Figure 6(b).

By simple derivation as given by equation (5), we can find that *g*_*i*_ is equal to *p*_*c*_ ⊕ *p*_*i*_. For a smooth block, all pixel values are close to each other. Therefore, there are a lot of zeros in the output image.

(5) $$\begin{array}{c} g_{i}=c_{i}⊕c_{c}=\left(p_{i}⊕K\right)⊕\left(p_{c}⊕K\right)=p_{i}⊕p_{c},\;i=1,2,\ldots ,8. \end{array}$$

After preprocessing, we apply the histogram shifting technique to embed secret data. According to the required embedding capacity, a threshold of gray level *g*_*th*_ is determined and the histogram is expanded by

(6) $$\begin{array}{c} g_{i}^{\prime }=\left\{\begin{array}{cc} g_{i}\times 2, & g_{i}<g_{th},\\ g_{i}+g_{th}, & g_{i}\geq g_{th}\text{ and }g_{i}<128,\\ g_{i}, & g_{i}\geq 128+g_{th}. \end{array}\right. \end{array}$$

A vacating band of width *g*_*th*_ after the gray level 128 is created. Then, the first *g*_*th*_ gray levels are shifted to even values without disrupting their order and the gray levels are shifted outward between *g*_*th*_ and 128. The threshold value *g*_*th*_, recorded with six bits, and the information in the vacating band are encoded and stored as metadata.

The binary secret stream is encrypted using *Key-III* with the conventional stream ciphering technique into an encrypted bitstream *S*={*b*_1_, *b*_2_, *b*_3_,…, *b*_*N*_}. For all embeddable pixels with *g*_*i*_′ < 2 × *g*_*th*_, we collect them in ascending order of gray level and in a raster scan order for pixels of the same gray level. Then, we consecutively embed secret bit by

(7) $$\begin{array}{c} {\hat{g}}_{i}=g_{i}^{\prime }+b_{j}. \end{array}$$

After embedding, postprocessing with the same operation as preprocessing is executed again to reverse the effect. For each block,

(8) $$\begin{array}{c} {\hat{g}}_{i}^{\prime }={\hat{g}}_{i}⊕{\hat{g}}_{c},\;i=1,2,\ldots ,8, \end{array}$$

where the definitions of ${\hat{g}}_{c}$ and ${\hat{g}}_{i}$ can refer to Figure 5.

To achieve reversibility of the proposed scheme, the histogram band in the range 128 ≤ *g*_*i*_ < 128+*g*_*th*_ erased by the vacating process of histogram shifting should be recorded. Since only a very small amount of data is required to record, we design a simple and straightforward coding rule. Six bits are used to record *g*_*th*_; twelve bits are used to record the total number of coded pixels; 3 bytes for each pixel are used to record its gray level *g*_*i*_ and coordinates (*x*, *y*) in the image. The image encryption and data embedding process is summarized as follows.

 
**Input:** cover image, binary secret stream, encryption key: *Key-I, Key-II,* data hiding key: *Key-III*
 
**Output:** encrypted image with data embedded
  Content owner:
 
**Step 1:** encrypt the image by block permutation with *Key-I* and stream ciphering with *Key-II*
  Data hider:
 
**Step 2:** preprocess the encrypted image according to equation (4)
 
**Step 3:** apply histogram shifting to vacate embedding area by equation (6)
 
**Step 4:** encode the erased histogram band into metadata
 
**Step 5:** collect the embeddable pixels in ascending order of gray level and raster scan order
 
**Step 6:** apply stream ciphering to the secret binary stream with *Key-III* into an encrypted data stream
 
**Step 7:** embed metadata first and then encrypted data stream by equation (7)
 
**Step 8:** postprocess the embedded image by equation (8) to produce the output image

The tiny image example given in Figure 5(c) is applied to illustrate the data embedding process as shown in Figure 7. The two encrypted image blocks are shown in Figure 7(a). The preprocessed blocks are shown in Figure 6(b), where we apply the threshold gray level *g*_*th*_=4 and the embeddable pixels are denoted by red characters. The embedding order of all embeddable pixels is labeled with green Arabic numerals. Except for the center pixel of each block, all pixel values are expanded according to equation (6). Then, the encrypted secret stream is embedded in the predefined order by equation (7) to obtain Figure 7(c). Finally, the two blocks are postprocessed to get Figure 7(d). An example of pixel processing is also given in the figure.

### 3.3. Data Extraction and Image Recovery Phase

The data extraction and cover image recovery are executed in the reverse order of encryption and embedding. The overall process is summarized as follows (Figure 8).

The data extraction and image recovery process.

**Input:** encrypted image with data embedded, encryption key: *Key-I*, *Key-II*, data hiding key: *Key-III.*
**Output:** binary secret stream, cover image.
Receiver:
**Step 1:** preprocess each block of the input image by
  (9) $$\begin{array}{c} {\hat{g}}_{i}={\hat{g}}_{i}^{\prime }⊕{\hat{g}}_{c},\;i=1,2,\ldots ,8, \end{array}$$
where the notation definitions of ${\hat{g}}_{c}$ and ${\hat{g}}_{i}^{\prime }$ are the same as equation (9).
**Step 2:** collect the first six pixels belonging to {0,1} in the raster scan order and convert them to get *g*_*th*_.
**Step 3:** according to *g*_*th*_, collect all embeddable pixels in the ascending order of ${\hat{g}}_{i}/2$ and raster scan order for the pixels of the same value, where ⌊·⌋ is the floor function.
**Step 4:** consecutively extract the metadata and encrypted secret stream by even-odd decision.
**Step 5:** decipher the binary secret stream using *Key-III.*
**Step 6:** backward shift the pixel values and recover the vacating band according to the metadata. The backward shifting is given by
  (10) $$\begin{array}{c} g_{i}=\left\{\begin{array}{cc} \left\lfloor \frac{{\hat{g}}_{i}}{2}\right\rfloor ,\; & {\hat{g}}_{i}<2\times g_{th},\\ {\hat{g}}_{i}-g_{th}, & {\hat{g}}_{i}\geq 2\times g_{th}\text{ and }{\hat{g}}_{i}<128+g_{th},\\ {\hat{g}}_{i}, & {\hat{g}}_{i}\geq 128+g_{th}. \end{array}\right. \end{array}$$
where ⌊·⌋ is the floor function.
**Step 7:** postprocess each block by
  (11) $$\begin{array}{c} c_{i}=g_{i}⊕c_{c},\;i=1,2,\ldots ,8, \end{array}$$
where the notation definitions of *c*_*c*_ and *g*_*i*_ are the same as equation (4).
**Step 8:** decipher the histogram recovered image using *Key-II.*
**Step 9:** apply backward permutation to obtain a cover image using *Key-I.*

The data embedded tiny illustrative image in Figure 7(d) is applied as an input of the data extraction and image recovery process as shown in Figure 7(a). The two blocks are preprocessed to get Figure 7(b). Then, according to *g*_*th*_=4, the secret data stream can be extracted, and the histogram can be recovered as shown in Figure 7(c). Next, we postprocess the two blocks to get Figure 7(d). Finally, we use the encryption key to decipher the image blocks. Note that we do not show the extraction of metadata and recovery of vacated histogram band as in an actual application.

## 4. Blockchain-Based Reversible Data Hiding System

The proposed blockchain system is presented in this section, with the aim of providing integrity and traceability in existing RDHEI. A consortium blockchain system is used in this paper, in which the participants in the blockchain network are trusted parties. For instance, the hospitals and health research institute (HRI) can form a consortium blockchain to share the medical images among themselves. In this way, an expensive consensus algorithm (e.g., PoW) is not required; it can be replaced with a lightweight algorithm like PBZT. Moreover, consortium blockchain is also a more appropriate choice as we do not expect any unauthorized person to join the blockchain network and gain access to the medical information, which is supposed to be private.

### 4.1. Architecture of the Proposed Blockchain-Based Reversible Data Hiding System

Figure 9 shows the architecture of the proposed blockchain system, which can be used to exchange medical images safely. Doctor A first encrypts the medical records of a patient and then generates the CSMI using the proposed RDHEI scheme, wherein the encrypted medical records are embedded into the patient's medical image. The encrypted medical records and CSMI are stored in the database of his hospital (Hospital X). A transaction block is generated and added to the blockchain.

With the proposed blockchain system, anyone who wants to share medical information can verify the integrity of transmitted data at the receiver end. For instance, Doctor A shares the CSMI with Doctor B and Medicate Institute Y. Upon receiving the CSMI, Doctor B first computes the hash value of received data and compares it against the blockchain to verify its integrity. He then extracts the hidden medical records with a legitimate key and then decrypts the medical records with another legitimate key. A similar process is performed by Medical Institute Y. The details on how to generate a new block and verify the integrity of CSMI are presented in the next section.

### 4.2. Process of Generating New Blocks and Verifying the Integrity of CSMI

Referring to Figure 10, the medical records of a patient are first encrypted by a symmetric key algorithm through the following equation:

(12) $$\begin{array}{c} C_{\text{MR}}=\text{Enc}\left(K_{1},\text{MR}\right), \end{array}$$

where MR refers to the medical records, *K*_1_ is the symmetric key, and *C*_MR_ is the resultant ciphertext. Next, we generate another key *K*_2_* *= *Key-I || Key-II || Key-III*, where *Key-I*, *Key-II*, and *Key-III* are the keys used in the proposed RDHEI scheme. We embed the encrypted medical records (*C*_MR_) into the medical image and generate a CSMI through the proposed RDHEI scheme. In Step 3, the generated CSMI and the hash value of the previous block in blockchain (*H*_prev_) are concatenated. The hash value of the current block is generated through the following equation:

(13) $$\begin{array}{c} H_{\text{curr}}=\text{Hash}\left(H_{\text{PREV}}||\text{CSMI}\right), \end{array}$$

where Hash can be any standardized cryptographic hash function (e.g., SHA-2 and SHA-3) and *H*_curr_ is the hash value of the current block. The newly generated block is transmitted to the blockchain network for the consensus process, wherein a lightweight algorithm can be used. Once the peers in the blockchain network approved the current block, a new block is generated (Step 5) and is added to the existing blockchain (Step 6). Assume that a person receives CSMI*′* from a legitimate member in the blockchain network. To verify the integrity of the received CSMI, he first computes the hash value: *H*_curr_′=Hash(*H*_PREV_*||*CSMI) following the same hash function used in the block creation process. Then, he compares *H*_curr_′ against the hash value *H*_curr_ stored in the blockchain. If both values are the same, then CSMI*′* is untampered; otherwise, CSMI*′* or *C*_MR_ has been modified.

The proposed blockchain system can be implemented with any popular blockchain framework, e.g., Hyperledger Fabric and Ethereum. Step 1 can employ an industry-grade block cipher (e.g., AES) to perform the encryption, while Step 2 can be carried out by using the techniques described in Section 3. Subsequently, Steps 3–6 are common operations found in a standard blockchain framework, which can be implemented easily.

### 4.3. Security Analysis

In this section, a security analysis on the proposed blockchain system is provided, with consideration of various attacking scenarios.

1. Attackers cannot retrieve the steganography of medical images. In the proposed system, the CSMI is stored in the database of the hospital. Assuming that the malicious attacker has access to the CSMI, he cannot recover the steganography of medical images (SMI). This is because he does not hold K2 to successfully recover the SMI. On top of that, he can never extract the patient's medical records embedded into CSMI
2. The proposed system can protect the confidentiality of medical records. The patient's medical records are being encrypted by a symmetric key algorithm with key *K*_1_, before embedding it into the medical image. Assume that the malicious attacker has access to the CSMI, and he had successfully extracted the SMI. In such a situation, he cannot successfully extract the medical records, because he does not have the *K*_1_ to decrypt them. Hence, the confidentiality of the patient's medical records is protected
3. The proposed system can achieve integrity. It is also possible that the malicious attacker is interested in creating fake CSMI instead of extracting information from it. For instance, one can generate fake keys *K*_1_′ to encrypt the legitimate medical records (*C*_MR_′) and then embed them to the other medical image to produce a fake CSMI′. This fake CSMI′ is being stored in the database as a new entry. However, the hospital can detect this fake CSMI′ easily by comparing it against the hash value stored in our blockchain system. Since CSMI′ is calculated from fake keys *K*_1_′ and *K*_2_′, the hash value generated (*H*_curr_′) is not the same as the one stored in the blockchain (*H*_curr_). In order to create fake CSMI′ that everyone trusts, the attacker needs to modify the blockchain accordingly. However, referring to equation (13), the hash value in each new block depends on the previous block. To modify one record in blockchain, the attacker must also recalculate all the subsequent blocks, which is almost impossible. Hence, the proposed system is secure against malicious attacks that attempt to compromise its integrity
4. The image encryption scheme is robust under chosen-plaintext analysis. The permutation process with *Key-I* has corrupted the block correspondence between the cover image and the encrypted image. Without the mapping information between the image blocks before and after encryption, chosen plaintext analysis is useless. Even if the block mapping is known, it is still too complicated for analysis since image blocks are encrypted with distinct keys generated by *Key-II*

## 5. Experimental Results and Discussion

In this section, we present the experimental results of the proposed RHDEI and its application to medical images. The hardware resources are Intel ® Core ™ i7-3770 CPU @ 3.40 GHz and 8 GB RAM PC. The application software is MATLAB R2017a running with Windows 10 Professional operating system. Six standard test images (see Figure 11) including “Airplane,” “Baboon,” “Boat,” “Lena,” “Peppers,” and “Sailboat” are applied to demonstrate the effectiveness of our scheme. The encrypted images are shown in Figure 12. The preprocessed images and postprocessed images with data embedded are given in Figures 13 and 14, respectively.

The histograms of the test images and their corresponding encrypted images are given in Figures 15 and 16. Referring to Figure 16, the histogram of encrypted images is evenly distributed in the entire range of gray levels regardless of the different image features. This indicates a high-security level of the proposed image encryption scheme.

The histogram after the preprocess of the embedding phase is given in Figure 17. For smooth images, the histogram is more concentrated while it is more distributed for complex images such as “Baboon.” Note that the histogram band of [128,192] gray levels is very “clear” by observation. To know the details, we further restrict the display range of the vertical axis to [0,200] pixels as shown in Figure 18. There are some pixels distributed in the band. To achieve the complete reversibility of the embedding scheme, the metadata includes three data segments. The first segment records the threshold *g*_*th*_ with six bits. The second segment records the number of pixels in the vacating band with twelve bits. The last segment contains all details of each pixel in the vacating band by one byte for its gray level and two bytes for its coordinates in the image. Therefore, the total length of metadata is 6+12+(3 × 8 × *N*_*p*_), where *N*_*p*_ is the number of pixels in the vacating band. After histogram shifting and data embedding, the histogram in Figure 17 changes to the distribution shown in Figure 19, where the applied threshold of vacating band is *g*_*th*_=64.  Figure 20 shows the resulting histogram of the marked encrypted image after postprocessing. The histogram is still evenly distributed and preserves at a high-security level.

Since the total number of pixels in the vacating band is very small, we can recover the histogram in a more efficient way by retrieving the first two segments of metadata to get *g*_*th*_ and determine the remaining length of metadata to be discarded. Thus, the recovery of the vacating band can be skipped, and the process is proceeded directly to extract the secret data stream. To know the visual quality of the approximated image, we apply the peak-signal-to-noise ratio (PSNR) index given by

(14) $$\begin{array}{c} \text{MSE}=\frac{1}{W\times H}\sum_{i=1}^{W}\sum_{j=1}^{H}{\left(I_{i,j}-I_{i,j}^{\prime }\right)}^{2}, \end{array}$$

(15) $$\begin{array}{c} \text{PSNR}=10\;\log_{10}\frac{255^{2}}{\text{MSE}}, \end{array}$$

where MSE is the mean square error between the cover image *I*_*i*,*j*_ and the approximated image *I*_*i*,*j*_′ and *W* and *H* are the width and height of the image. The second measure of similarity between them is the structural similarity (SSIM) defined by

(16) $$\begin{array}{c} \text{SSIM}\left(I,I^{\prime }\right)=\frac{\left(2\mu_{I}\mu_{I^{\prime }}+c_{1}\right)\left(2\sigma_{II^{\prime }}+c_{2}\right)}{\left(\mu_{I}^{2}+\mu_{I^{\prime }}^{2}+c_{1}\right)\left(\sigma_{I}^{2}+\sigma_{I^{\prime }}^{2}+c_{2}\right)}, \end{array}$$

where *μ*_*I*_, *μ*_*I*′_, *σ*_*I*_, and *σ*_*I*′_ are the mean values and standard deviations and *σ*_*II*′_ is the covariance of the two images.

The experimental results of the proposed RDHEI scheme with different thresholds are listed in Table 1. The “capacity” and “metadata” are measured in bits. The actual embedding capacity of secret data can be calculated by subtracting the amount of metadata from the “capacity” value. The “ER” is the embedding rate measured in bits per pixel (bpp). The PSNR and SSIM values listed in the table indicate that the approximated images under fast recovery have good visual quality.

Figure 21 shows the PSNR values with respect to the embedding rate (ER). The threshold value determines the width of the vacating band and therefore degrades the visual quality. However, the ER also increases with the increased threshold. Another important point of observation is that the PSNR value is dependent on the image feature. The most complex image “Baboon” has the lowest PSNR level among all.

The second set of test images are two medical images downloaded from the website of MIDAS/National Alliance for Medical Image Computing (NAMIC) as shown in Figure 22. The image size 256 × 256 is relatively smaller than the standard test images in the first experiment. The encrypted images, preprocessed images, and postprocessed images are given in Figures 23–25, respectively. Histograms of the cover images are shown in Figure 26. Notice that the pixel values are concentrated to very low gray levels due to the inherent nature of MRI images. This phenomenon is especially beneficial to our data hiding scheme. The histogram distributions for different processing phases are given in Figures 27–31. The experimental values are listed in Table 2. The major difference from the first experiment is that the embedding rate reaches 0.6 bpp at the lowest threshold of *g*_*th*_=4, which is much higher than the capacity of standard test images. At the highest threshold of *g*_*th*_=64, the medical images can reach an embedding rate of 0.8 bpp.

Figure 32 compares the proposed scheme with other related works, including VRAE-based schemes (Zhang et al.'s scheme [9, 12]) and VRBE-based schemes (Cao et al.'s scheme [21] and Malik et al.'s scheme [22]), for two typical test images “Lena” and “Baboon.” Note that all these schemes are completely reversible. The PSNR values are compared under the situation of discarding some information in image deciphering. The proposed scheme reaches a good embedding rate with a good visual quality of the approximation image. The scheme proposed in [17] is VRBE-based; therefore, it provides only one fixed embedding rate.

Compared to a recently proposed RDH technique by Anushiadevi et al. [23], the proposed technique offers a flexible threshold (*g*_*th*_) to allow performance tuning. The user can flexibly select a higher embedding capacity or higher PSNR by adjusting *g*_*th*_; this is not found in [23]. Another recent work that offered homomorphic encryption on RDH was proposed by Anushiadevi et al. [24]. Our proposed technique shows performance on par with them in terms of ER, PSNR, and flexible threshold configuration.

## 6. Conclusion

Medical images are important assets to the medical industry, and they should be protected to avoid potential infringement of privacy. To achieve this goal, we propose an RDHEI scheme, in which the cover image is encrypted by block permutation using encryption *Key-I* and stream ciphering using encryption *Key-II*. Then, the encrypted patient data is embedded into the encrypted image through *Key-III* to produce a secure CSMI. Experimental results show that the performance of the proposed RDHEI scheme is excellent when applied to medical images. The embedding rate is over 0.8 bpp for typical medical images. An image of high visual quality can be recovered even if the receiver only holds the image encryption keys. Since most processes of the proposed RDHEI scheme are based on the simple Exclusive-OR operation, our scheme can be executed very efficiently. To provide an integrity check, we propose a blockchain system on top of the RDHEI. The hash value of CSMI is stored in a commonly used blockchain system for future verification. The proposed RDHEI blockchain system allows the user to check the integrity of CSMI from time to time, which shows additional benefit compared to the conventional RDHEI schemes.

## Figures and Tables

**Figure 1:** Blockchain data structure.

**Figure 2:** The RDHEI scheme proposed by Zhang et al. [9].

**Figure 3:** The proposed RDHEI scheme.

**Figure 4:** An illustrative example of block permutation.

**Figure 5:** An illustrative example of block permutation and stream ciphering.

**Figure 6:** Pixel labeling of an encrypted block and its corresponding output after preprocessing. (a) Pixel labeling of a block and (b) output of preprocessing.

**Figure 7:** An illustrative example of the proposed image encryption and data embedding process.

**Figure 8:** An illustrative example of the proposed data extraction and image recovery process.

**Figure 9:** Architecture of the proposed blockchain system.

**Figure 10:** Transaction flow of the proposed blockchain system.

**Figure 11:** Cover images of size 512 × 512. (a) Airplane. (b) Baboon. (c) Boats. (d) Lena. (e) Peppers. (f) Sailboat.

**Figure 12:** The encrypted images. (a) Airplane. (b) Baboon. (c) Boats. (d) Lena. (e) Peppers. (f) Sailboat.

**Figure 13:** Preprocessed images. (a) Airplane. (b) Baboon. (c) Boat. (d) Lena. (e) Peppers. (f) Sailboat.

**Figure 14:** Postprocessed images with data embedded. (a) Airplane. (b) Baboon. (c) Boats. (d) Lena. (e) Peppers. (f) Sailboat.

**Figure 15:** Histogram of cover images. (a) Airplane. (b) Baboon. (c) Boat. (d) Lena. (e) Peppers. (f) Sailboat.

**Figure 16:** Histogram of encrypted images. (a) Airplane. (b) Baboon. (c) Boat. (d) Lena. (e) Peppers. (f) Sailboat.

**Figure 17:** Histogram of preprocessed images. (a) Airplane. (b) Baboon. (c) Boat. (d) Lena. (e) Peppers. (f) Sailboat.

**Figure 18:** Histogram of preprocessed images at a finer scale. (a) Airplane. (b) Baboon. (c) Boat. (d) Lena. (e) Peppers. (f) Sailboat.

**Figure 19:** Histogram of data embedded images before postprocessing. (a) Airplane. (b) Baboon. (c) Boat. (d) Lena. (e) Peppers. (f) Sailboat.

**Figure 20:** Histogram of postprocessed (final) images. (a) Airplane. (b) Baboon. (c) Boat. (d) Lena. (e) Peppers. (f) Sailboat.

**Figure 21:** Performance comparisons of test images with the proposed scheme.

**Figure 22:** Cover images of size 256 × 256. (a) Medical image A. (b) Medical image B.

**Figure 23:** The encrypted images. (a) Medical A. (b) Medical B.

**Figure 24:** Preprocessed images. (a) Medical A. (b) Medical B.

**Figure 25:** Postprocessed images with data embedded. (a) Medical A. (b) Medical B.

**Figure 26:** Histogram of cover images. (a) Medical A. (b) Medical B.

**Figure 27:** Histogram of encrypted images. (a) Medical A. (b) Medical B.

**Figure 28:** Histogram of preprocessed images. (a) Medical A. (b) Medical B.

**Figure 29:** Histogram of preprocessed images at a finer scale. (a) Medical A. (b) Medical B.

**Figure 30:** Histogram of data embedded images. (a) Medical A. (b) Medical B.

**Figure 31:** Histogram of postprocessed images. (a) Medical A. (b) Medical B.

**Figure 32:** Comparisons of the proposed scheme with related works for typical test images. (a) Lena. (b) Baboon.

**Table 1:** Experimental results of the proposed scheme with different thresholds.

Image	Metrics	*g*_*th*_ = 4	*g*_*th*_ = 8	*g*_*th*_ = 16	*g*_*th*_ = 32	*g*_*th*_ = 64
Airplane	Capacity	102125	140358	171658	190931	202715
	Metadata	42	66	162	6666	12858
	ER (bpp)	0.38	0.53	0.65	0.72	0.77
	PSNR	61.64	58.29	54.77	37.72	34.35
	SSIM	0.9999	0.9999	0.9999	0.995	0.9912
Baboon	Capacity	30506	56047	93320	134879	173447
	Metadata	1242	2298	4962	12810	51138
	ER (bpp)	0.11	0.21	0.35	0.51	0.66
	PSNR	42.61	40.32	36.99	32.79	26.12
	SSIM	0.999	0.9983	0.9961	0.9895	0.9516
Boat	Capacity	79348	119982	153134	184078	209831
	Metadata	114	210	546	1866	10626
	ER (bpp)	0.3	0.45	0.58	0.7	0.8
	PSNR	56.36	52.21	46.9	40.83	32.5
	SSIM	0.9999	0.9999	0.9996	0.9983	0.9879
Lena	Capacity	83908	127070	164152	194295	209334
	Metadata	138	162	354	738	4506
	ER (bpp)	0.32	0.48	0.62	0.74	0.79
	PSNR	53.11	52.07	48.24	45.27	36.04
	SSIM	0.9999	0.9999	0.9997	0.9993	0.9944
Pepper	Capacity	81892	127696	167267	195067	214845
	Metadata	258	498	954	1794	5586
	ER (bpp)	0.31	0.48	0.63	0.74	0.81
	PSNR	51.15	47.48	43.9	40.5	35.82
	SSIM	0.9998	0.9997	0.9993	0.9982	0.9944
Sailboat	Capacity	56910	93681	134503	176246	195452
	Metadata	474	930	1794	3906	10122
	ER (bpp)	0.21	0.35	0.51	0.67	0.74
	PSNR	45.23	41.76	39.11	35.87	31.43
	SSIM	0.9995	0.999	0.998	0.9958	0.9872

**Table 2:** Experimental results of the MRI medical images with different thresholds.

Image	Metrics	*g*_*th*_ = 4	*g*_*th*_ = 8	*g*_*th*_ = 16	*g*_*th*_ = 32	*g*_*th*_ = 64
Medical A	Capacity	39671	43490	48507	52655	56038
	Metadata	66	114	234	738	1554
	ER (bpp)	0.6	0.66	0.74	0.8	0.85
	PSNR	70.1	57.02	42.68	37.44	35.34
	SSIM	0.9999	0.9999	0.9989	0.9971	0.9953
Medical B	Capacity	40608	43388	46851	50168	53448
	Metadata	138	258	546	1122	4338
	ER (bpp)	0.61	0.66	0.71	0.76	0.81
	PSNR	49.6	45.67	41.45	37.48	30.82
	SSIM	0.9999	0.9996	0.999	0.9976	0.9871

## Data Availability

The data used in the experiments and discussions in the paper are available within this article.
